# Optimization of the Purifying Process for Columbianetin-*β*-D-Glucopyranoside from *Angelicae Pubescentis* Radix and Evaluation of Its Analgesic Activity Using Hot Plate Test

**DOI:** 10.1155/2021/9944270

**Published:** 2021-08-04

**Authors:** Yaqian Zhang, Yuqiao Yang, Ye Shang, Chunxiao Liang, Jun He, Jin Li, Yanxu Chang

**Affiliations:** ^1^Tianjin State Key Laboratory of Modern Chinese Medicine, Tianjin University of Traditional Chinese Medicine, Tianjin 300193, China; ^2^Tianjin Key Laboratory of Phytochemistry and Pharmaceutical Analysis, Tianjin University of Traditional Chinese Medicine, Tianjin 300193, China

## Abstract

The objective of this work was to provide an economic and practical method for the purification of columbianetin-*β*-D-glucopyranoside from *Angelicae Pubescentis* Radix extract. In the static adsorption and desorption, the effects of resin type (D101, HP-20, AB-8, GDX-201, and DA201), contact time (10–360 min), and temperature (298–318 K) were assessed on columbianetin-*β*-D-glucopyranoside adsorption efficiency in laboratory. GDX-201 resin showed the best adsorption and desorption properties for columbianetin-*β*-D-glucopyranoside. The kinetic data revealed that the equilibrium time for columbianetin-*β*-D-glucopyranoside adsorption was achieved within 150 min. Moreover, the adsorption kinetic curve was well in accordance with the pseudo-second-order equation (*R*^2^ > 0.99). The rate controlling step of the adsorption process was the intraparticle diffusion. The Langmuir isotherm models (*R*^2^ > 0.99) could describe the whole adsorption process, which was exothermic and spontaneous according to the result of thermodynamics tests. In the dynamic adsorption and desorption process, the optimum loading flow (4, 5, and 6 BV/h), ethanol concentration (0–60%), and elution volume (10–230 mL) were optimized. Under optimal conditions of 4 BV/h loading flow, 6.7 BV loading volume, 25% ethanol, and 14 BV elution volume, the content of columbianetin-*β*-D-glucopyranoside in the product was increased 29.61-fold from 0.45% to 13.32 ± 0.64% with yield of 88.03 ± 2.76% by an experiment of lab-scale enlargement. Then, columbianetin-*β*-D-glucopyranoside was further purified by PHPLC and its purity was more than 98%. Additionally, the analgesic activity of the columbianetin-*β*-D-glucopyranoside was assessed by hot plate test. The experimental results showed that columbianetin-*β*-D-glucopyranoside significantly increased the latency of pain response in mice. This study demonstrated columbianetin-*β*-D-glucopyranoside could be as a potentially natural analgesic component. It could be summed up that the established method was successfully applied to purifying columbianetin-*β*-D-glucopyranoside from *Angelicae Pubescentis* Radix extract.

## 1. Introduction

*Angelicae Pubescentis* Radix (APR), the dried roots of *Angelica pubescens* Maxim. f. *biserrata* Shan et Yuan, is mainly distributed in Sichuan and Hubei provinces in China. As a time-honored traditional Chinese medicine, it has been extensively used to treat arthralgia and rheumatism [1]. Coumarins are the major active ingredients, and the modern pharmacology has confirmed that it has anti-inflammatory, analgesic pharmacological activity [2–4]. Columbianetin-*β*-D-glucopyranoside (CBG) is one of coumarin compounds found in APR which has been proven to have the prevention platelet aggregation and protection against glutamate-induced toxicity [5, 6]. In our previous study, we had found that CBG (Figure 1) could move through the blood-brain barrier of SD rats and mainly excrete through faecal path [7]. In order to further study the pharmacology activity of coumarins and control the quality of TCMs, a simple and efficient enrichment and purification method is urgently required. Therefore, much focus needs to be placed on the extraction and separation of coumarins in TCMs.

In the extraction process, it is relatively difficult to obtain the extract merely containing the required compounds, which means that an excellent postextraction method is needed to acquire the compounds of interest. The heating reflux extraction coupled with silica gel column method was usually used to extract and purify coumarin ingredients from Traditional Chinese Medicine [8, 9]. Nevertheless, this method is not suitable for industrial scale-up production due to low recovery, being time-consuming, great waste of organic reagents, and environmental pollution. Comparatively speaking, macroporous adsorption resins (MARs) have been widely used to purify compounds from food and TCMs because of their numerous superiorities, such as low cost, high adsorbance, easy regeneration performance, and being environmentally friendly [10–12]. Accordingly, MARs may be applied as adsorbents for the separation and purification of CBG from the APR extract. However, there was no report on the purification of CBG from APR by using MARs. Moreover, its analgesic effect assessment was yet to be reported. Hot plate test is a classic model for screening analgesics due to its excellent advantages, including less damage to tissues and simple operation [13]. Hence, hot plate test was used to evaluate analgesic effect of CBG.

The aim of the present research was to investigate the potential use of macroporous resin as adsorbent for the enrichment of CBG from APR extract. The adsorption mechanism was systematically investigated using different models, including the adsorption/desorption behaviors, kinetics, isotherms, and thermodynamics. Furthermore, in the process of dynamic adsorption and desorption, the optimum loading flow and ethanol concentration/volume on the enrichment of CBG onto MARs were optimized. Moreover, the enriched fraction was further separated and purified by PHPLC. On this basis, a hot plate method was established to evaluate CBG analgesic effect. The findings contribute to the MAR selection for CBG or other coumarins separation from TCMs and guide the larger-scale CBG purification for medical applications.

## 2. Materials and Methods

### 2.1. Chemicals and Reagents

Standard of CBG (purity ≥98% on HPLC) was separated and purified from APR in our laboratory (Tianjin, China). Analytical-grade ethanol and chromatographic-grade acetonitrile were provided by Concord Science Co. Ltd. (Tianjin, China). Deionized water was obtained from a Milli-Q Academic water system (Millipore, Milford, MA, USA). All of macroporous adsorbent resins were purchased from Welch Materials Inc. (Shanghai, China).

### 2.2. Preparation of Crude Extracts

*Angelicae Pubescentis* Radix was obtained from Bozhou city (Anhui, China). Simply, 2 kg of APR was extracted by using the heating reflux method for 2 h. The specific conditions were as follows: solid-liquid ratio, extract solution, and extract times were 1 : 10, 70% ethanol, and three times, respectively. The final extract was concentrated and dried, and the sample was placed at −20°C for further use.

### 2.3. HPLC Analysis of CBG

CBG was analyzed using an Agilent 1200 HPLC system equipped with VWD detection. All the samples' concentration was detected with the detection wavelength of 325 nm on an Agilent Zorbax Eclipse XDB-C18 (4.6 × 250 mm, 5 *μ*m). The mobile phase comprised acetonitrile (A) and water (B) using the following elution conditions: 0–12 min, 22–22% A; 12–15 min, 22%–95% A; 15–21 min, 95–100% A; 21–23 min, 100–22% A; and 23–28 min, 22–22% A. The mobile phase flow rate was chosen as 1 mL/min and the injection volume was set at 10 *μ*L. The column temperature was set at 30 °C. The linear equation was *y* = 25.883*x* + 2.194 (*R*^2^ = 0.9998), where *y* was peak area and *x* was the concentration of CBG.

### 2.4. Selection of Macroporous Resins

The static adsorption and desorption properties of different resins on APR extracts were investigated to obtain the best resin. In brief, 0.5 g of resin was added to 20 mL of sample solution and shocked at 120 rpm for 6 h at 298 K. The resins were rinsed with deionized water after the adsorption equilibrium was reached. Next, the resins were eluted with 20 mL of 95% ethanol. The concentrations of CBG in adsorption equilibrium and desorption solution were determined by HPLC. The adsorption capacity, desorption capacity, and desorption ratio of the five tested resins were figured up using the following formulas.

Adsorption capacity is as follows:

(1) $$\begin{array}{c} Q_{e}=\frac{\left(C_{0}-C_{e}\right)V_{i}}{W}. \end{array}$$

Desorption capacity is as follows:

(2) $$\begin{array}{c} Q_{d}=\frac{C_{d}V_{d}}{W}. \end{array}$$

Desorption ratio is as follows:

(3) $$\begin{array}{c} D=\frac{C_{d}V_{d}}{\left(C_{0}-C_{e}\right)Vi}, \end{array}$$

where *Q*_*e*_ and *Q*_*d*_ are the adsorption and desorption capacities (mg/g); *C*_0_, *C*_*e*_, and *C*_*d*_ stand for the original, balance, and desorption concentration of CBG in the sample solution, respectively (*μ*g/mL); *V*_*i*_ and *V*_*d*_ are the volumes of the original and desorption sample (mL); *W* represents the weight of dry resin (g).

### 2.5. Adsorption Isotherm and Adsorption Thermodynamics

The isotherm for the adsorption of CBG onto GDX-201 resin was performed at different temperatures (298, 308, and 318 K). First, 0.5 g of the resin and 20 mL sample solution were added to a 100 mL conical flask. Second, the conical flask was shaken (120 rpm) at different temperatures (298, 308, and 318 K) for 6 h. Then, HPLC 1200 was used to determine the concentration of CBG. To further analyze the adsorption process, the tests data of adsorption isotherm were fitted with Langmuir equation and Freundlich isotherm model.

The Langmuir equation is as follows:

(4) $$\begin{array}{c} \frac{C_{e}}{Q_{e}}=\frac{1}{K_{L}Q_{m}}+\frac{C_{e}}{Q_{m}}. \end{array}$$

Separation factor is as follows:

(5) $$\begin{array}{c} R_{L}=\frac{1}{1+K_{L}C_{0}}. \end{array}$$

The Freundlich model is as follows:

(6) $$\begin{array}{c} Q_{e}=K_{F}e^{1/n}, \end{array}$$

where *Q*_*m*_ stands for the largest adsorbance (mg/g); *K*_*L*_ is the equilibrium constant of the Langmuir model; *K*_*F*_ is the Freundlich constant; and 1/*n* is an empirical constant indicating the adsorption intensity of the adsorbent.

Adsorption thermodynamics are used to further clarify the change of adsorption energy and adsorption mechanism. Entropy, enthalpy, and Gibbs energy were obtained using the following formulas:

(7) $$\begin{array}{c} \Delta G=-RT\;\ln\text{ K},\\ \ln\text{ K}=-\frac{\Delta H}{RT}+\frac{\Delta S}{R}, \end{array}$$

where *T* and *R* stand for the absolute temperature (K) and the gas constant (8.314 J/mol·K), respectively.

### 2.6. Adsorption Kinetics

First, 0.5 g of GDX-201 resin and 20 mL of APR extract (the concentration of CBG is 477.58 *μ*g/mL) were transferred into a 100 mL beaker flask. Then, the flask was shaken (120 rpm) at 298 K for 6 h, and the concentrations of CBG during the adsorption process were determined at regular intervals (10, 20, 30, 40, 50, 60, 90, 120, 150, 180, 240, 300, and 360 min). To better comprehend the adsorption process, the five following models were applied for analyzing the adsorption kinetics data.

The pseudo-first-order model is as follows:

(8) $$\begin{array}{c} Q_{t}=Q_{e}\left(1-e^{-K1t}\right). \end{array}$$

The pseudo-second-order model is as follows:

(9) $$\begin{array}{c} \frac{1}{Q_{t}}=\frac{1}{Q_{e}^{2}K_{2}t}+\frac{1}{Q_{e}}. \end{array}$$

The intraparticle diffusion model is as follows:

(10) $$\begin{array}{c} Q_{t}=K_{i}t^{1/2}+C. \end{array}$$

The liquid film diffusion model is as follows:

(11) $$\begin{array}{c} -\ln\left(1-\frac{Q_{t}}{Q_{e}}\right)=K_{3}t, \end{array}$$

where *Q*_e_ is the adsorption capacity at equilibrium and *Q*_t_ is the adsorption capacity at any time (mg/g).

### 2.7. Dynamic Adsorption and Desorption Tests

In order to get the best purification condition, both dynamic adsorption and desorption tests were executed with a glass column wet-packed with the GDX-201 resin (10 mm × 400 mm, 1 BV = 15 mL). The dynamic adsorption tests were carried out by feeding APR extract solution (477.58 *μ*g/mL) at different flow rates (4, 5, and 6 BV/h), and the optimal adsorption speed was screened on the foundation of the adsorbance of the GDX-201 resin column for CBG. The dynamic desorption tests were carried out by using ultrapure water (5 BV) to wash the GDX-201 resin columns firstly and then eluted by using 5%–60% ethanol (5 BV) at a speed of 4 BV/h, respectively, and the optimal ethanol solution concentration was chosen based on desorption ratio of the CBG. Whereafter, to optimize the volume of desorption ethanol solution, the sample-fed GDX-201 resin columns were desorbed by using the optimized concentration at a speed of 4 BV/h.

### 2.8. Enrichment of CBG by GDX-201 Resin

The compound of the CBG was separated and enriched on glass columns (40 mm × 600 mm, 1 BV = 215 mL) wet-packed with GDX-201 macroporous resin. A total of 1000 mL of APR extract solution (the concentration of CBG is 477.58 *μ*g/mL)was absorbed by the GDX-201 resin column at a flow rate of 4 BV/h. After reaching the adsorption equilibrium, the impurities of sample were firstly removed by using ultrapure water (10 BV) and 5% ethanol (10 BV), and then 25% ethanol (14 BV) was applied to elute CBG from the GDX-201 resin column at a flow rate of 4 BV/h. Finally, the CBG fraction was obtained from the 25% ethanol elution solution that was concentrated and dried by using a rotary evaporator with vacuum dryer.

### 2.9. Separation of CBG by PHPLC

After enrichment with GDX-201 resin, CBG was further purified at a flow rate of 9 mL/min on a Shimadzu Prominence LC-20 AP PHPLC (Tokyo, Japan) equipped with Agilent Eclipse XDB-C18 (250 × 21.2 mm, 7 *μ*m) column. The mobile phase consisted of water (A) and acetonitrile (B). The gradient method was as follows: 0–20 min, 22–22% B; 20–25 min, 22–100% B; and 25–35 min, 100% B. The final injection volume was 1.0 mL and the detection wavelength was 325 nm.

### 2.10. In Vivo Hot Plate Test in Mice Assay

The hot plate test was carried out to assess the analgesic performance of mice after oral administration of CBG according to the method reported previously [14]. Female C57BL/6 mice (20 ± 2 g) were obtained from Beijing HFK Biotechnology Co., Ltd. All animal experiments were carried out in strict accordance with the experimental animal guidelines. Animal welfare was authorized by the animal ethics committee of Tianjin University of Traditional Chinese Medicine. CBG (25, 75, 125 mg/kg), 0.5% CMC-Na (10 mL/kg), and aspirin (75 mg/kg) were orally administered to mice before the test. Then, the mice were placed on top of thermostatic hot plate (55 °C). The reaction latency period was recorded as the time taken for the mice to respond to the heat stimulation by licking their paw. In order to avoid damage to the tissues of mice paw, the maximum pain threshold was set to 45 s. The maximum possible analgesia (MPA) was calculated using the following equation:

(12) $$\begin{array}{c} \text{MPA}=\frac{\text{HPT}-\text{HPC}}{45-\text{HPC}}\times 100\%, \end{array}$$

where HPT stands for hot plate latency for treatment (s) and HPC stands for hot plate latency for 0.5% CMC-Na (s).

### 2.11. Statistical Analysis

All data were shown as mean ± standard deviation values. The error bars in all figures represent the standard deviation of triplicates. Statistical analysis was carried out by Origin 2018 (OriginLab, Northampton, Massachusetts, USA) and GraphPad Prism 5.0 software (GraphPad, San Diego, California, USA). Significant differences between variables were measured by one-way ANOVA, and differences were regarded as significant when *P* < 0.05.

## 3. Result and Discussion

### 3.1. Screening of the Optimum Resin

The differences of adsorption capacity, desorption capacity, and desorption ratio of CBG from APR extract by five resins (D101, HP-20, AB-8, GDX-201, and DA201) were investigated (Table 1). Compared with the other four resins, GDX-201 resin had better adsorption capacity (9.01 ± 0.08 mg/g) and the highest desorption ratio (98.13 ± 2.60%). This may be due to the existence of poly(divinylbenzene) in its structure. Hence, GDX-201 resin was chosen to purify CBG. Besides, as a polar resin, DA-201 resin had better adsorption performance (7.44 ± 0.48 mg/g) than other resins, like D101, HP-20, and AB-8 resin. This phenomenon can be explained by similar compatibility rules.

### 3.2. The Effect of Contact Time/Temperature on CBG Adsorption Capacity

In order to study the effect of contact time on the adsorption capacity of GDX-201 resin, experiments were conducted at different contact time (10–360 min).  Figure 2 shows the effect of contact time on CBG adsorption capacity on GDX-201 resin at 298 K. The adsorption capacity of CBG on GDX-201 resin increased rapidly in the first 60 min. In the following time, the growth rate was slow, and the adsorption equilibrium was reached after 150 min. This phenomenon may be explained by the large available surface area of the resin at the beginning, but it decreases rapidly until it reaches equilibrium with the increase in time.

The effect of temperatures on adsorption ratio of GDX-201 resin was also investigated.  Figure 3 shows the effect of temperature on CBG adsorption ratio on GDX-201 resin. With the temperature increasing from 298 to 318 K, the adsorption ratio gradually decreased. This result indicated that the lower temperature could promote GDX-201 resin for the CBG adsorption. The reason for this phenomenon may be that, with the increase of temperature, the adsorption between the active sites of the adsorbent decreases, and the trend of CBG desorption from the interface to the solution increases.

### 3.3. Adsorption Dynamics

The study on adsorption kinetics plays a crucial role for the technological design. The four adsorption kinetic equation parameters of CBG on GDX-201 resin are displayed in Table 2. According to the degree of correlation coefficient (*R*^2^) close to 1, it can be judged that the adsorption process of CBG on GDX-201 resin can be described by pseudo-second-order model, and its *R*^2^ is greater than 0.99 (0.9908).

The slowest step called the rate-controlling step controls the rate of the whole process, while a process is made up of many successive steps, whether chemical or physical. As a general rule, the speed of the slowest step has a positive correlation with the speed of the whole reaction to a certain extent. The two steps of liquid film diffusion and intraparticle diffusion were used to describe the solid-liquid adsorption process. It is particularly essential to predict the rate-controlling step in the adsorption process to understand the mechanism of the adsorption. The linear relationship between the liquid film diffusion model and the intraparticle diffusion model and time can be used to determine the rate-controlling steps of the adsorption process. The results are shown in Figures 4(c) and 4(d) and Table 2. There was a good linear relationship between −ln(1 − *q*_*t*_/*q*_*e*_) and *t* (*R*^2^ > 0.98), yet it does not pass through the origin, indicating that liquid film diffusion is the main controlling step in the initial stage of adsorption instead of the only controlling step (Figure 4(c) and Table 2). It is worth noting that although the intraparticle diffusion kinetic model does not fit the entire adsorption process well (*R*^2^ = 0.7631), the process can be divided into 3 stages (Figure 4(d)). The first stage was called liquid film diffusion from 10 to 30 min (*R*^2^ = 0.9988). At this stage, the spherical macroporous resin adsorbent was encapsulated in a layer of liquid film, and the adsorbate can be adsorbed on the surface of the resin through the liquid membrane. The second stage, called intraparticle diffusion, occurred in 40–120 min (*R*^2^ = 0.9852). The adsorption equilibrium process in 150–360 min (*R*^2^ = 0.9827) was the third stage. At this stage, the concentration of CBG in the aqueous solution decreased and the available adsorption sites were reduced. Simultaneously, the intraparticle diffusion became slower, and the concentration of sample solution was basically unchanged, so the third stage had little effect on the rate of the entire adsorption process [15–17]. In summary, the intraparticle diffusion time was longer (about 80 min), which was 4 times than that of the first stage (about 20 min). Therefore, intraparticle diffusion was the rate-controlling step of this adsorption process.

### 3.4. Adsorption Isotherm and Adsorption Thermodynamics

Adsorption isotherm was usually applied to understand the effect of temperature on resins' adsorption capacity. In this study, the adsorption isotherms of CBG on GDX-201 resin were investigated at 298, 308, and 318 K. As shown in Figure 5(a), as the balance concentration of CBG increased, the balance adsorbance of GDX-201 resin for CBG increased. Besides, the equilibrium adsorption capacity of CBG on the GDX-201 resin decreased with increased temperature, which showed that the lower temperature could promote the adsorption of GDX-201 resin for CBG. Langmuir and Freundlich models were used to describe the adsorption isotherms, which are shown in Figures 5(b) and 5(c); and the fitting parameters are summarized in Table 3. The adsorption isotherms of CBG on the GDX-201 resin were well fitted by Langmuir model (*R*^2^ > 0.99). It indicated that the adsorption process of CBG on GDX-201 resin might be monomolecular adsorption. The value of *R*_*L*_ stands for unfavorable (*R*_*L*_ > 1), linear (*R*_*L*_ = 1), favorable (0 < *R*_*L*_ < 1), and nonreversible (*R*_*L*_ = 0) adsorption process [18]. The values of *R*_L_ were between 0.092 and 0.129 in the experimental concentration range, indicating that the adsorption of GDX-201 resin for CBG was a preferential procedure. For the Freundlich isotherm model, 1/*n* is an empirical constant indicating the adsorption intensity of the adsorbent. It is believed that 1/*n* greater than 0 and less than 0.5 indicates being easy to absorb [19]. In the present study, the values of 1/*n* were 0.2439–0.2657, which suggested that the GDX-201 resin has good adsorption performance for CBG.

According to the slope and intercept in the linear relationship between lnK and 1/*T* (Figure 5(d)), the thermodynamics equation parameters for CBG on GDX-201 resin at different temperature are calculated and presented in Table 4. The Gibbs energy (∆*G*) values were between −27.03 and −26.10 kJ/mol. The negative Gibbs energy (∆*G*) values showed that the adsorption was feasible and spontaneous, and the enhancement of ∆*G* negative values with decrease of temperature indicates that lower temperature was beneficial to the adsorption process. The value of enthalpy (∆*H*) was less than 0 (−14.74 kJ/mol), which indicated that the adsorption of CBG on the GDX-201 resin is an exothermic process. Besides, the absolute value of ∆*H* was below 43 kJ/mol, which suggested that the adsorption of CBG by GDX-201 resin belongs to physical adsorption process [20–22]. The value of entropy (∆*S*) was 41.51 J/mol, which revealed that the adsorption of CBG on the resin is a random enhancement process.

### 3.5. Dynamic Adsorption and Desorption

Generally, dynamic leak curves were investigated at different speeds (4, 5, and 6 BV/h) for obtaining the optimal speed and sample loading volume. It can be seen from Figure 6(a) that a lower flow (4 BV/h) resulted in the increment of CBG adsorption capacity due to sufficient contact between CBG and the resin matrix. Although the high flow rate could save time, the corresponding actual adsorption capacity was reduced. Hence, 4 BV/h was chosen as appropriate feeding flow rate, and the corresponding feeding volume was about 6.7 BV (100 mL). Dynamic desorption was executed by using the gradient elution method at a flow rate of 4 BV/h. The desorption capacity increased with increasing ethanol concentration. When the ethanol content reached 25%, the desorption ratio was the highest (Figure 6(b)). Therefore, 25% ethanol was used to enrich CBG from GDX-201 resin column. As shown in Figure 6(c), CBG was completely eluted from GDX-201 resin column when the volume of 25% ethanol reached 14 BV. Comparing the chromatograms of crude extract with those after treatment, it was obvious that CBG became the mainly high peak (Figures 7(a) and 7(b)). Besides, it can be reflected clearly that the adsorption ratio of the GDX-201 resin was maintained above 90% by five consecutive cyclic adsorption experiments, indicating that the GDX-201 resin could be used for enrichment of CBG from APR extract (Figure 6(d)).

### 3.6. Enrichment of CBG by GDX-201 Resin and PHPLC

As shown in Table 5, the content of CBG was increased 32.63-fold from 0.45% to 14.68 ± 0.84% with a recovery yield of 90.44 ± 1.03%, when the feed volume was 100 mL. Through the scale-up experiment, the content of CBG was increased 29.61-fold from 0.45% to 13.32 ± 0.64% with a recovery yield of 88.03 ± 2.76%. These results further showed that GDX-201 resin could be used to enrich CBG on a large scale from APR extract.

To further increase the content of CBG, the PHPLC was used (Figure 7(c)). Finally, 1013.2 mg of CBG was obtained from 25% ethanol fraction; and the purity of CBG was over 98% (Figure 7(d)).

### 3.7. Comparison of the MARs Method with Other Methods in the Purification of Coumarins in TCMs

A comparison of the proposed MARs method and other separation methods to purify the coumarins of TCMs is shown in Table 6. It was clearly observed that although multiple coumarin components were separated in these reported studies, the eluent systems were complex, and the organic solvents such as petroleum ether, ethyl acetate, n-hexane, and methanol were highly toxic and were not easy to recycle in HSCCC. It indicated that these processes were complex and not suitable for scale-up production. More importantly, in the present study, we used the macroporous resin as adsorbent for the enrichment of CBG. Ethanol as an environmentally friendly organic solvent, which is easy to recover and recycle, was used as the elution solvent to desorb CBG from GDX-201 resin in this study. Hence, the MARs method is simple, efficient, and environmentally friendly for separation and purification of the coumarin constituents from APR; and the method developed in the present study is easier to scale up purified coumarins.

### 3.8. In Vivo Hot Plate Test in Mice Assay

The analgesic activity assay of CBG was tested using hot plate test. As shown in Figure 8, the positive control group (75 mg/kg aspirin) could significantly enhance the reaction time of the hot plate after administration. At medium concentration (75 mg/kg), CBG could significantly increase the reaction time of the hot plate at 60 (*P* < 0.05), 90 (*P* < 0.05), 120 (*P* < 0.05), and 240 min (*P* < 0.01) after oral treatment. At high concentration (125 mg/kg), CBG could significantly increase the reaction time of the hot plate at 30 (*P* < 0.05), 60 (*P* < 0.05), 90 (*P* < 0.05), 120 (*P* < 0.05), and 240 min (*P* < 0.01) after oral treatment. In order to see further difference in the analgesic potential between CBG and aspirin, the MPA percentage of the two substances was calculated (Figure 9). After 240 min of administration, the MPA of CBG (75 mg/kg and 125 mg/kg) exceeded that of aspirin, which further indicated that CBG had analgesic activity.

## 4. Conclusions

A simple and efficient method for purification of columbianetin-*β*-D-glucopyranoside from APR extract with macroporous resins was successfully established. Among the five resins, the GDX-201 resin displayed the best adsorption and desorption capacity for CBG. The adsorption kinetic experimental data of CBG on the GDX-201 resin could be well fitted by the pseudo-second-order equation (*R*^2^ > 0.99). Langmuir model (*R*^2^ > 0.99) gave a better fit compared to Freundlich model. Thermodynamic test results showed that the adsorption process of CBG on the GDX-201 resin was exothermic and spontaneous. The intraparticle diffusion was the rate-controlling step of the adsorption process. Then, under the dynamic optimal conditions, the content of columbianetin-*β*-D-glucopyranoside in the product was increased 29.61-fold from 0.45% to 13.32 ± 0.64% with yield of 88.03 ± 2.76%. The purity of the product reached 98% after purification by PHPLC.

The result demonstrated that the isolation method was useful and simple, showing a prospect for industrial-scale purification of CBG from APR extract in the future. In addition, our research indicated that CBG increased the latency to pain response in hot plate test. In summary, columbianetin-*β*-D-glucopyranoside could be used as a potential analgesic drug.

## Figures and Tables

**Figure 1:** Chemical structure of columbianetin-*β*-D-glucopyranoside.

**Figure 2:** The effect of contact time on adsorption capacity of GDX-201 resin (resin dose = 25 mg/mL, CBG concentration = 477.58 *μ*g/mL, and temperature = 298 K).

**Figure 3:** The effect of temperatures on adsorption ratio of GDX-201 resin (resin dose = 25 mg/mL, CBG concentration = 477.58 *μ*g/mL, and contact time = 150 min).

**Figure 4:** (a) Pseudo-first-order model. (b) Pseudo-second-order model. (c) Liquid film diffusion model. (d) Intraparticle diffusion model of CBG on GDX-201 resin at 298 K.

**Figure 5:** (a) Adsorption isotherms. (b) Langmuir model. (c) Freundlich model. (d) Plot of lnK versus 1/*T* for the estimation of thermodynamic parameters of CBG on GDX-201 resin at different temperature.

**Figure 6:** (a) Dynamic leakage curve; (b) gradient elution curve; (c) desorption curve of CBG on an GDX-201 resin column 150 mL (10 BV), H_2_O; 150–300 mL (10 BV), 5% ethanol; 300–510 mL (14 BV), 25% ethanol; (d) the relationship between the cycle numbers and the adsorption ratio.

**Figure 7:** HPLC chromatograms of the sample: (a) before treatment and (b) after treatment by the GDX-201 resin; (c) by PHPLC; (d) CBG purified by PHPLC.

**Figure 8:** Analgesic effects of CBG in the hot plate test in mice. Effects of different doses of CBG and aspirin on reaction latency of mice in the hot plate (55°C) at different times after administration (*n* = 10 per group). ^*∗*^*P* < 0.05 and ^*∗∗*^*P* < 0.01 compared to vehicle-treated mice.

**Figure 9:** Maximum possible analgesia (MPA).

**Table 1:** Physical properties and adsorption/desorption capacity of five test macroporous resins.

Resins	Structure	Polarity	Particle size (mm)	Surface area (m^2^/g)	Adsorption capacity (mg/g)	Desorption capacity (mg/g)	Desorption ratio (%)
D101	Polystyrene	Nonpolar	0.30–1.25	480–550	3.18 ± 0.05	2.38 ± 0.02	74.96 ± 0.73
AB-8	Polystyrene	Weakly polar	0.30–1.25	480–520	3.48 ± 0.05	2.73 ± 0.14	78.34 ± 1.10
HP-20	Polystyrene	Nonpolar	0.30–1.25	550–600	3.09 ± 0.07	2.23 ± 0.17	72.16 ± 1.17
DA-201	Polystyrene	Polar	0.30–1.25	≧200	7.44 ± 0.48	7.04 ± 0.23	94.87 ± 4.72
GDX-201	Poly(divinylbenzene)	—	0.30–1.25	510	9.01 ± 0.08	8.84 ± 0.07	98.13 ± 2.60

**Table 2:** Adsorption kinetics parameters of CBG on GDX-201 resin at 298 K.

Kinetics model	Parameters	CBG
Pseudo-first-order	*Q*_*e*_ (mg·g^−1^)	8.7821
	*K*_1_ (min^−1^)	0.0494
	*R* ^2^	0.8931

Pseudo-second-order	*Q*_e_ (mg·g^−1^)	9.3721
	*K*_2_ (g·mg^−1^·min^−1^)	0.0093
	*R* ^2^	0.9908

Liquid film diffusion	*K*_3_	0.0207
	*R* ^2^	0.9878

Intraparticle diffusion (10–360 min)	*I* (mg·g^−1^)	5.2058
	*K*_*i*_ (mg·g^−1^·min^−0.5^)	0.2562
	*R* ^2^	0.7631

Intraparticle diffusion (10–30 min)	*I* (mg·g^−1^)	1.4153
	*K*_*i*_ (mg·g^−1^·min^−0.5^)	0.9659
	*R* ^2^	0.9988

Intraparticle diffusion (40–120 min)	*I* (mg·g^−1^)	4.6772
	*K*_*i*_ (mg·g^−1^·min^−0.5^)	0.3863
	*R* ^2^	0.9852

Intraparticle diffusion (150–360 min)	*I* (mg·g^−1^)	8.5831
	*K*_*i*_ (mg·g^−1^·min^−0.5^)	0.0291
	*R* ^2^	0.9827

**Table 3:** Langmuir and Freundlich parameters for CBG on GDX-201 resin.

Temperature (K)	Langmuir equation				Freundlich equation		
	*R* ^2^	*K*_*L*_	*Q*_*m*_ (mg/g)	*R*_*L*_	*R* ^2^	*K*_*F*_	1/*n*
298	0.9997	134.13	9.32	0.092	0.8190	13.66	0.2439
308	0.9997	121.22	9.17	0.101	0.8507	13.56	0.2548
318	0.9996	92.08	9.05	0.129	0.8568	13.38	0.2657

**Table 4:** Thermodynamics equation parameters for CBG on GDX-201 resin.

Temperature (K)	∆G (kJ/mol)	∆H (kJ/mol)	∆S (J/mol)
298	−27.03	−14.74	41.51
308	−26.78		
318	−26.10		

**Table 5:** Results of separation of CBG on columns packed with GDX-201 resin.

GDX-201 resin (g)	Feed volume (mL)	Before purification (%)	After purification (%)	Recovery (%)	Enrichment of multiple
3	100	0.45	14.68 ± 0.84	90.44 ± 1.03	32.63
30	1000		13.32 ± 0.64	88.03 ± 2.76	29.61

**Table 6:** Comparison of the MARs method with other methods in the purification of coumarins in TCMs.

No.	Purification compounds	Source	Type of solvent	Method	Reference
1	Xanthotoxin, isopimpinellin, bergapten, imperatorin, and osthole	*Cnidium monnieri* (L.) Cusson	Light petroleum–ethyl acetate–methanol–water	HSCCC^a^	[23]
2	Xanthotoxin, isopimpinellin, bergapten, imperatorin, and osthole	*Cnidium monnieri* (L.) Cusson	*n*-Hexane–ethyl acetate–ethanol–water	HSCCC^a^	[24]
3	Xanthotoxin, bergapten, columbianetin acetate, osthole, isoimperatorin, and columbianadin	*Angelicae Pubescentis* Radix	*n*-Hexane–ethyl acetate–methanol–water	CCC-PHPLC^b^	[25]
4	Columbianetin-*β*-D-glucopyranoside	*Angelicae Pubescentis* Radix	Ethanol–water	MARs^c^	This work

^a^High-speed countercurrent chromatography. ^b^Countercurrent chromatography and preparative liquid chromatography. ^c^Macroporous resins.

## Data Availability

All the datasets presented in this study are included in the article.
